The article "ALKBH5 Is Lowly Expressed in Esophageal Squamous Cell Carcinoma and Inhibits the Malignant Proliferation and Invasion of Tumor Cells" was retracted in 2023. Reasons: signs of a paper mill; compromised peer review; unreliable results or conclusions.

# ALKBH5 Is Lowly Expressed in Esophageal Squamous Cell Carcinoma and Inhibits the Malignant Proliferation and Invasion of Tumor Cells

**DOI:** 10.1155/2021/1001446

**Published:** 2021-11-28

**Authors:** Jinqiu Li, Hongqiang Liu, Shanglin Dong, Yunbo Zhang, Xiao Li, Jing Wang

**Affiliations:** ^1^Department of Radiotherapy, The First Affiliated Hospital of Hebei North University, Zhangjiakou, 075000 Hebei, China; ^2^Department of Ultrasonography, The First Affiliated Hospital of Hebei North University, Zhangjiakou, 075000 Hebei, China; ^3^Department of Medical Imaging, The First Affiliated Hospital of Hebei North University, Zhangjiakou, 075000 Hebei, China; ^4^Department of Oncology, Zibo Bashan Wanjie Hospital, Zibo, 255213 Shandong, China; ^5^Life Science Research Center, Hebei North University, Zhangjiakou, 075000 Hebei, China

## Abstract

**Background:**

Modification of N^6^-methyladenosine (m^6^A) and RNA m^6^A regulatory factors is required in cancer advancement. The contribution of m^6^A and its alteration in esophageal squamous cell carcinoma (ESCC) is still unclear.

**Results:**

ALKBH5 was lowly expressed in ESCC tissues, which the total m^6^A level was increased in ESCC tissue than the presentation in normal healthy tissue. The pcDNA3.1-ALKBH5 recombinant plasmid was transfected into KYSE-150 and Eca-109 cells. The overexpression of ALKBH5 is responsible for a significant reduction of the total m^6^A levels in Eca-109 and KYSE150 cells, inhibiting the proliferation capability, migration, and cell invasion.

**Conclusions:**

ALKBH5 as a demethylase was lowly expressed in cancer progression of ESCC and acts as a crucial component in ESCC progression.

## 1. Background

Esophageal cancer (EC) ranks seventh in the global cancer incidence rate and sixth cause of cancer mortalities, globally [1]. Two leading pathological conditions of EC are squamous cell carcinoma (ESCC) or skin cancer and adenocarcinoma (EAC) or distal esophagus cancer, which have significantly different risk factors, geographic distribution, and treatment strategies. In China, EC accounts for the majority of cancer mortalities, among which ESCC is the leading subtype (80%) [2]. China's ESCC cases account for half of the burden of the global ESCC patients and more than 90% of Asia's [3]. Its patients are generally diagnosed as advanced [4]. At present, the survival rate in ESCC cases is still very low [5].

N^6^-Methyladenosine (m^6^A) is referred to as a modification of RNA in mammals [6]. m^6^A is edited by the complex of methyltransferase (“writers,” METTL3/METTL14/WTAP/RBM15/ZC3H1/KIAA1429) and cleared by demethylase (“erasers,” ALKBH5, and FTO). “Readers” (YTHDF1/2/3, YTHDC1/2, HNRNPA2/B1, HNRNPC, HNRNPG, eIF3, IGF2BP1/2/3, and Prrc2a) can selectively recognize m^6^A modified RNA and perform specific biological functions. Modification of m^6^A initiates RNA metabolism, which includes RNA degradation, transportation, positioning, and translation [7, 8].

Xu et al. construct a prognostic mark composed of HNRNPC and ALKBH5, the development that the prognostic mark can act as an independent prognostic marker [9]. Moreover, Guo et al. identify the prognostic characteristics of EC patients including ALKBH5 and HNRNPA2B1 [10].

In this research, we will clarify the function of ALKBH5 in the malignant growth and invasion of ESCC cells *in vitro*.

## 2. Results

### 2.1. ALKBH5 Is Lowly Expressed in ESCC

First, the presentation of gene expression of ALKBH5 was measured in 23 ESCC tissue samples using qRT-PCR and IHC.  Figure 1(a) shows the relative mRNA levels of ALKBH5 which was lowly expressed in ESCC tissues, i.e., *P* < 0.05. The results of IHC showed that ALKBH5 had abundant protein expression in normal esophageal tissues (Figure 1(b)). However, the gene expression of ALKBH5 protein was significantly reduced in ESCC tissues (Figures 1(b) and 1(c)). The data statistics indicted that ALKBH5 was highly expressed in 78.26% (18/23) of normal and healthy esophageal tissues, but only highly expressed in 39.13% (9/23) of ESCC patients' tissues (Figure 1(c), *P* < 0.05). Adding that, the total m^6^A levels in ESCC were detected by ELISA (Figure 1(d)). The total m^6^A level in ESCC was higher compared to the normal esophageal tissue (Figure 1(d), *P* < 0.05). In summary, there was a significant increase of total m^6^A levels seen in ESCC tissues, and the expression of ALKBH5 was significantly decreased compared with normal esophageal tissues.

### 2.2. Proliferation Inhibition of ESCC Cells by ALKBH5

pcDNA3.1-ALKBH5 plasmid (OE) was transfected into ESCC cells, and the function-gain experiments were performed. As seen in Figure 1(e), ALKBH5 was markedly overexpressed in Eca-109 and KYSE150 cells following transfection of the pcDNA3.1-ALKBH5 plasmid (*P* < 0.05). In addition, the overexpression of ALKBH5 significantly reduced the total m^6^A levels (Figures 2(a) and 2(b)). Regarding the ESCC cells and its proliferation, both CCK-8 (Figure 2(c)) and clone formation (Figure 2(d)) assays suggested that ALKBH5 inhibited the ESCC cell proliferation and its growth.

### 2.3. Apoptosis Induction of ESCC Cells by ALKBH5

Apoptosis signals are responsible for regulating the proliferation of tumor cells. Therefore, the impact of ALKBH5 overexpression on the signals of apoptosis of Eca-109 and KYSE150 cells was detected. Flow cytometry indicated that after overexpression of ALKBH5, the apoptotic cell ratio increased significantly, the Bax expression and cleaved caspase3 increased, and Bcl2 expression decreased (Figures 3(a) and 3(b)). In summary, ALKBH5 overexpression induced the apoptosis signals in ESCC cells.

### 2.4. Motility Inhibition of ESCC Cells by ALKBH5

The migration and invasion of Eca-109 and KYSE150 cells transfected with the pcDNA3.1-ALKBH5 plasmid were explained. As shown in Figure 4(a), the invasion cell numbers of both transfected with the pcDNA3.1-ALKBH5 plasmid were obviously decreased. Furthermore, the overexpression of ALKBH5 significantly reduced the migration cell numbers in ESCC cells (Figures 4(b)–4(d)).

## 3. Discussion

m^6^A modification and RNA m^6^A regulatory factors contribute to cancer progression. Among them, certain m^6^A regulatory factors have been found to be significantly related to the progression and prognosis of ESCC. For example, METTL3 is highly expressed in ESCC and significantly relates to the patient prognosis [11]. Furthermore, the overexpression of METL3 promotes the proliferation and invasion of ESCC cells [12]. Zhang et al. detect the gene expression proportion of m^6^A-related proteins in 348 ESCC tissues by using ELISA and find that the expressions of METTL3 and METTL14 in ESCC pathological tissues are significantly upregulated, while the expressions of FTO and ALKBH5 are significantly downregulated, compared with normal tissues. It is consistent with our research detected in 23 ESCC tissue samples using RT-qPCR and IHC. This study also detected the total m^6^A level in ESCC tissues by using ELISA. Consistent with the expression level of m^6^A regulatory factors, the total m^6^A level in ESCC tissues increased significantly.

However, Xu et al. analyze the RNA transcriptome data of 161 EC samples and 11 normal tissue samples in the TCGA database and find no significant differential expression of FTO and ALKBH5 [9]. This result may be affected by the pathological subtype of tumor tissue samples or the lack of normal tissue samples. However, they still find the prognostic signal consisting of HNRNPC and ALKBH5 based on this cohort. In addition, Liu et al. find a significantly high expression of gene FTO by the ESCC tissue microarray [13]. ALKBH5, as a homologue of FTO [14], works with FTO to maintain the balance of levels of m^6^A in the transcriptome [15]. This result seems to be contrary to our research. However, our study failed to detect the expression level and mechanism of FTO.

Genetic dissimilarity of m^6^A modifier genes is possibly linked to ESCC risk. The rs2416282 of YTHDC2 promoter is identified as significantly connected with ESCC risk [16]. This allele specifically affects the binding of transcription factors. In addition, knocking down the YTHDC2 expression significantly inhibits the proliferation of ESCC cells [16]. However, Xu et al. analyze the genetic mutations in the TCGA EC cohort through the cBioPortal database [9]. The results show that the genetic variation frequency of YTHDF1, ZC3H13, and KIAA1429 is 7-8%, and the most common variation is amplification. The frequency of other adjustment factors is less than 3%. They believe that the changes in the gene expression levels of these regulatory factors are not caused by genetic changes.

This study demonstrates the use of pcDNA3.1 plasmid to overexpress ALKBH5 protein and found that ALKBH5 contributes to suppressing cancer. Our study reported the contribution of ALKBH5 expression to altering the biological functionality of human cells of ESCC *in vitro*. These outcomes point out that ALKBH5 is involved in the malignant growth and aggressive response of ESCC.

## 4. Conclusions

Concluding this, ALKBH5 as a demethylase is lowly expressed in ESCC tissues. ALKBH5 regulates the total m^6^A level of ESCC cells and contributes as a vital entity in ESCC progression. However, we have not explored the expression and role of ALKBH5 homologue FTO, nor have we disclosed the molecular process that regulates the downregulation of ALKBH5 expression in ESCC tissues.

## 5. Methods

### 5.1. Patients and Tissue Samples

This study recruited 23 ESCC patients who were diagnosed and received surgical resection without neoadjuvant/adjuvant treatment. The tissue samples were confirmed pathologically after resection.

### 5.2. Cell Culture and Transfection

KYSE-150 and Eca-109 cell lines were used to execute this study. The selected cell bank to obtain these cell lines was the Chinese Academy of Sciences. RPMI 1640 medium was used to culture these cell lines with supplementation of 10% FBS. The culture conditions are 5% CO_2_ and 37°C. ALKBH5 cDNA synthesization was performed and cloned into pcDNA3.1 expression vector. Subsequently, the cell transfection of recombinant plasmid was carried out by the Lipofectamine 2000 reagent.

### 5.3. RT-qPCR

Total RNA from tissues or cells transfected with recombinant plasmid for 24 h was extracted and synthesized into cDNA. GADPH is an internal reference, and the relative expression level of ALKBH5 was calculated using the 2^-∆∆CT^ method.

### 5.4. Immunohistochemistry Staining Analysis (IHC)

Tissue samples were formalin-fixed and paraffin-embedded. The paraffin samples were made into tissue sections with a thickness. The tissue segments underwent deparaffinization, rehydration, and microwave treatment. After blocking, the tissue segments were incubated with ALKBH5 antibody (1 : 500, ab195377, rabbit monoclonal antibody, Abcam) and with a biotin-labeled secondary antibody. Staining was performed by the enhanced DAB chromogenic kit, and the tissue segments were dehydrated and fixed.

The score of each section was the product of the positivity proportion of stained cells (*R*) and the staining intensity score (*S*). *R* scores included 0 (<5%, negative), 1 (5-25%, occasional), 2 (25-50%, focus), and 3 (>51%, diffuse). *S* scores included 0 (negative), 1 (weak), 2 (medium), and 3 (strong). A score higher than 3 was considered a high expression of ALKBH5.

### 5.5. Total m^6^A Level Detection

Total m^6^A level detection was performed to measure the total m6A levels of tissue samples or cells transfected with recombinant plasmid for 24 h. For ELISA, the EpiQuik m^6^A RNA methylation quantification ELISA kit (P-9005-96, Epigentek) was used. For the dot blot assay, the TRIzol reagent separated total RNA, and the mRNA was separated and enriched by mRNA isolation systems of Polyattract® (A-Z5300, A&D Technology Corporation). After being exposed to UV light for 7 min, the mRNA was cross-linked with the optimized Amersham Hybond-N^+^ membrane. After washing with PBST buffer, the membrane was blocked with 5% skimmed milk and incubated with anti-m^6^A antibody, and the HRP Substrate of Immobilon Western Chemilum was used to stain (Merck Millipore).

### 5.6. Western Blot

Protein was solubilized by RIPA buffer, and SDS-PAGE gel electrophoresis was used for separation of protein bands and final transfer of protein bands to the PVDF membrane. 5% skimmed milk closed the membrane. Subsequently, the membrane was incubated with primary antibody and with the secondary antibody. The enhanced chemiluminescent HRP substrate (Menlo Park, CA) was used for the visualization of chemiluminescence.

### 5.7. Cell Proliferation Assays

For the CCK-8 assay, 2000 cells/well were seeded in a 96-well plate. After culturing for a certain period of time, the old medium was removed, and a new medium was added containing 10% CCK-8 reagent. The absorbance value of each well at wavelength of 450 nm was measured with the help of a microplate reader. To perform the colony formation assay, 1000 transfected cells were extracted and seeded in each microplate well of a 6-well plate, and cell culturing was performed for up to 2 weeks. The formed clones were stained with 0.1% crystal violet.

### 5.8. Flow Cytometry Detection

Trypsinization of cells was performed without adding EDTA and resuspended to 1 × 10^6^ cells/ml with binding buffer. FITC-Annexin V PI were added to the cell suspension. After mixing thoroughly, the FACScan flow cytometer system (BD Biosciences, San Jose, California) was used immediately for detection.

### 5.9. Mobility Assay

For the transwell assay, cells suspended in serum-free medium were added to the upper chamber. After the 24-hour duration, fixation of cells was performed; the cells were present at the bottom of the chamber membrane where 4% paraformaldehyde was used for cell fixation and crystal violet dye for cell staining. To perform the wound healing assay, a wound was created in the cell monolayer with the help of a cell scraper. The washing of sloughed cells was performed with PBS. After culturing for a specified time, pictures were taken and the wound healing rate was calculated.

### 5.10. Statistics

The data was analyzed with SPSS 20.0. Student's *t*-test and one-way ANOVA were used to test the difference between groups. *P* < 0.05 was considered statistically significant.

## Figures and Tables

**Figure 1:** ALKBH5 is lowly expressed in ESCC tissues. The mRNA (a) and protein (b) expression of ALKBH5 in 23 pairs of ESCC and adjacent normal tissue samples using qRT-PCR and IHC. (c) The data statistics of IHC. (d) The total m^6^A levels in ESCC and normal tissues by ELISA. (e) ALKBH5 protein was significantly overexpressed in Eca-109 and KYSE150 cells following transfection of the pcDNA3.1-ALKBH5 plasmid (OE). NC: negative control. *P* < 0.05.

**Figure 2:** ALKBH5 inhibits ESCC cell proliferation. The total m^6^A levels in Eca-109 and KYSE150 cells transfected with the pcDNA3.1-ALKBH5 plasmid (OE) by dot blot assays (a) and ELISA (b). The proliferation and growth of Eca-109 and KYSE150 cells transfected with the pcDNA3.1-ALKBH5 plasmid (OE) by CCK-8 (c) and colony formation (d) assays. NC: negative control. *P* < 0.05.

**Figure 3:** ALKBH5 induces ESCC cell apoptosis. (a) Flow cytometry detection for apoptosis of Eca-109 and KYSE150 cells transfected with the pcDNA3.1-ALKBH5 plasmid (OE). (b) The expression of apoptosis-related proteins by western blot. NC: negative control. *P* < 0.05.

**Figure 4:** ALKBH5 inhibits the ESCC cell migration and invasion. The invasion (a) and migration (b–d) of Eca-109 and KYSE150 cells transfected with the pcDNA3.1-ALKBH5 plasmid (OE) by transwell and wound healing assays. NC: negative control. *P* < 0.05.

## Data Availability

The datasets used and/or analyzed to conduct this study are available from the corresponding author on valid request.
